The article "MicroRNA expression profiling during the life cycle of the silkworm (Bombyx mori)" was retracted in 2011. Reason: duplicated images.

# MicroRNA expression profiling during the life cycle of the silkworm (*Bombyx mori*)

**DOI:** 10.1186/1471-2164-10-455

**Published:** 2009-09-28

**Authors:** Shiping Liu, Liang Zhang, Qibin Li, Ping Zhao, Jun Duan, Daojun Cheng, Zhonghuai Xiang, Qingyou Xia

**Affiliations:** 1 The Key Sericultural Laboratory of Agricultural Ministry, College of Biotechnology, Southwest University, Chongqing 400715, PR China; 2 National Engineering Center for Beijing Biochip Technology, Life Science Parkway, Changping District, Beijing 102206, PR China; 3 Beijing Genomics Institute at Shenzhen, Shenzhen 518083, PR China; 4 Beijing Institute of Genomics, Chinese Academy of Sciences, Beijing 100000, PR China; 5 Institute of Agricultural and Life Sciences, Chongqing University, Chongqing, 400030, PR China

## Abstract

**Background:**

MicroRNAs (miRNAs) are expressed by a wide range of eukaryotic organisms, and function in diverse biological processes. Numerous miRNAs have been identified in *Bombyx mori*, but the temporal expression profiles of miRNAs corresponding to each stage transition over the entire life cycle of the silkworm remain to be established. To obtain a comprehensive overview of the correlation between miRNA expression and stage transitions, we performed a whole-life test and subsequent stage-by-stage examinations on nearly one hundred miRNAs in the silkworm.

**Results:**

Our results show that miRNAs display a wide variety of expression profiles over the whole life of the silkworm, including continuous expression from embryo to adult (miR-184), up-regulation over the entire life cycle (let-7 and miR-100), down-regulation over the entire life cycle (miR-124), expression associated with embryogenesis (miR-29 and miR-92), up-regulation from early 3^rd ^instar to pupa (miR-275), and complementary pulses in expression between miR-34b and miR-275. Stage-by-stage examinations revealed further expression patterns, such as emergence at specific time-points during embryogenesis and up-regulation of miRNA groups in late embryos (miR-1 and bantam), expression associated with stage transition between instar and molt larval stages (miR-34b), expression associated with silk gland growth and spinning activity (miR-274), continuous high expression from the spinning larval to pupal and adult stages (miR-252 and miR-31a), a coordinate expression trough in day 3 pupae of both sexes (miR-10b and miR-281), up-regulation in pupal metamorphosis of both sexes (miR-29b), and down-regulation in pupal metamorphosis of both sexes (miR-275).

**Conclusion:**

We present the full-scale expression profiles of miRNAs throughout the life cycle of *Bombyx mori*. The whole-life expression profile was further investigated via stage-by-stage analysis. Our data provide an important resource for more detailed functional analysis of miRNAs in this animal.

## Background

MiRNAs are an abundant class of small (~22 nucleotides) noncoding RNAs expressed by a variety of eukaryotic organisms and viruses [1,2], which represent at least 1% of predicted genes within the genomes of individual species [3]. A mammalian genome may contain >500 genes encoding miRNAs [4,5]. Accumulating evidence shows that miRNAs function in a broad range of biological processes, including development, cellular differentiation, proliferation, metabolism and apoptosis [1,6-8]. Organisms devoid of miRNAs undergo arrest during development [9,10]. Recent studies additionally implicate miRNAs in the pathogenesis of human diseases, including cancer and metabolic disorders [11-15]. Moreover, miRNAs are required for normal steroid hormone signaling [16]. Interestingly, Dicer and miRNAs are not prerequisites for the development of zebrafish germline stem cells [17], despite being essential for zebrafish development [9]. However, in *Drosophila*, miRNA pathways appear essential for stem cell division and for bypassing the G1/S checkpoint of the cell cycle [18]. This dissimilarity may reflect diverse mechanisms in the proliferation and differentiation of pluripotent stem cells [19]. Computational predictions of miRNA targets indicate that these noncoding RNAs regulate hundreds of different mRNAs at the posttranscriptional level, and over 30% of animal genes [6,20]. However, to date, the roles of only a handful of known miRNAs have been experimentally determined. The current repression models of the mechanisms of miRNA-mediated gene silencing are still the subject of considerable debate [21], and many potential targets may actually be pseudotargets, thus preventing miRNAs from binding to their authentic targets via sequestration [22].

*B. mori*, the characteristic representative of lepidoptera, undergoes four distinctive main developmental stages, defined as embryo, larva, pupa, and adult moth. Silkworms have no characteristic feeding behavior at the adult stage, but display prominent traits, such as silk production, monophagy, and voltinism [23]. Therefore, *B. mori *is considered an important model organism to investigate various biological phenomena, including development, gene regulation, and morphological innovation [23]. Increasing numbers of miRNAs have been experimentally identified in the silkworm [24-27]. Several of these are temporally regulated or stage-specifically expressed, as observed by microarray analysis at four time-points [24]. However, the lifespan of the silkworm is over 50 days, with each of the four main metamorphosis stages lasting for several to more than 20 days. Therefore, examination of a few time-points is unlikely to reflect the accurate expression patterns of miRNAs over the entire life cycle of this animal [28]. Several heterochronic genes function in a regulatory pathway to influence the timing of cellular development, thereby ensuring a coordinated schedule of developmental events [29,30]. Correlation between miRNA expression and normal behavior is suggested in *Drosophila *adults [31]. In the present study, particular attention was focused on the detailed temporal profiling of miRNAs responding to developmental stage transitions of silkworms. The microarray data discussed in this publication have been deposited in NCBI's Gene Expression Omnibus [32] under accession number GSE18030 . The data revealed wide diversity in miRNA expression, ranging from stage-specific to constitutive patterns. Our study provides a broad overview of miRNA expression in the developing silkworm, and is thus an important initial step in elucidating the functions of miRNAs in this animal.

## Results

### General profile of miRNA expression over the whole life cycle of *Bombyx mori*

To determine the expression profiles of miRNAs in the developing silkworm, we performed microarray hybridization with 106 cDNA probes complementary to 92 miRNAs (see Additional file 1). Additional file 1 contains the main information, including mature and putative precursor sequences, foldback arms, 9× genome location data (site distribution, intergenic, intronic, or overlapping CDS; and chromosome), miRbase designation where available, and folding energy. All probes for miRNAs as well as negative and positive controls were printed in triplicate on the microarray slides (see Methods and Additional file 2). Half of the 92 miRNAs passed the filtering expression threshold, 35 were also confirmed by Northern blotting, and 15 (including bantam and miR-1) were robustly expressed from the embryo to adult stages (Additional files 3 and 4). The use of alternative probes for some miRNAs generally resulted in similar expression profiles (for example, in the case of miR-275# and miR-275), strongly confirming probe authenticity. Expression peaks for all established miRNAs were distributed over nine time-points. We observed up-regulation of 7 miRNAs and down-regulation of 10 miRNAs over the whole life cycle of the silkworm (Additional file 4). One new silkworm miRNA, miR-970, presented the highest signal on microarray at the early 1^st ^instar larva stage, which was confirmed by Northern blotting (Additional file 3). Four miRNAs (miR-281-5p, miR-281-3p, miR-79, and miR-317) were not detected until the silkworm hatched (eIL1), and were subsequently expressed at high levels until the birth of the adult moth, in microarray analysis (Additional file 4). miR-124 was typically down-regulated during silkworm development from day 6 embryo to adult moth, and undetectable after the 3^rd ^instar larva stage (Figure 1A, Additional file 4). In contrast, both microarray and Northern blotting analyses confirmed that let-7 and miR-100 were coordinately up-regulated, gradually accumulating from late 1^st ^molt until the 3^rd ^molt stage (Figure 1A, C, Additional file 4). These oscillations were coincident with the traditional watershed in sericulture management between the early larval and late larval stages. miR-29b displayed the highest expression at the embryo stage, and rapidly decreased in level after the 1^st ^molt larval stage, but rose significantly once more in fresh female moths carrying eggs in the abdomen (Figure 1A), raising the possibility of an involvement in oogenesis and embryogenesis. Interestingly, in other organisms, such as the mouse, miR-29b was almost undetectable in the embryo, but extensively expressed in the adult during brain development [33]. The expression patterns of miR-34b and miR-275 fluctuated in a complementary manner (Figure 1B). Specifically, miR-34b expression was restricted to instar larvae and adults, and was absent in the embryo, molt larvae, and pupae (Additional file 4). Ecdysone and *Broad-Complex *are responsible for the down-regulation of miR-34 in the development of *Drosophila *[34]. In fact, miR-34 is highly conserved, and its homologs have been widely identified in several other species across phyla. Recent studies show that members of this family, miRNA-34a-c, are direct transcriptional targets of p53, and participate in the suppression of cell proliferation [35,36]. In contrast to miR-34b, a faint expression signal from miR-275 was initially detected at early 3^rd ^molt, followed by slight up-regulation in early 4^th ^instar, early 4^th ^molt, and early 5^th ^instar larvae. This miRNA was highly expressed in early spinning larva and up-regulated to peak levels in the new pupa, but was remarkably absent in new female adults (Figure 1B). The expression profile derived from microarray data was supported by Northern blotting results (Figure 1C). Microarray analyses revealed that miR-92 was exclusively expressed at day 6 embryo, late 2^nd ^molt, and early pupal stages (Figure 1A), but strong expression was confirmed in day 6 embryos only by Northern blotting (Figure 1C). The miRNA profiles obtained with the general whole-life array provide an insight into the stage-specific miRNA transcriptome, and may thus facilitate the identification of sequential classes of miRNAs and their primary targets associated with distinct developmental stages.

**Figure 1:** **Temporal expression profile of miRNAs obtained with the whole-life test**. (A) Specific miRNAs were up-regulated or down-regulated over the entire life cycle of the silkworm. (B) Comparison of the expression profiles of miR-275 and miR-34b during the life cycle of silkworm. (C) Northern blotting analysis of miRNAs during the silkworm life cycle. 5srRNA and U6 were used as the loading controls.

### Expression profile of miRNAs in silkworm embryos

In the course of embryogenesis, large gene regulatory networks generate refined spatial and temporal patterns of expression [37]. Silkworm embryogenesis is initiated by formation of the zygote nucleus (synkaryon) within about 2 hours after egg deposition, and develops through diverse phases for about 10 days before hatching [38]. Only one time-point (day 6 embryo) was examined using the whole-life array, and this did not provide sufficient information on expression profiles in developing embryos of silkworm. We further assessed 9 and 11 time-points using microarray and Northern blotting, respectively, leading to significant extension of the range of temporal profiles of miRNA expression. In all, 36 unique miRNAs satisfied the expression standard for microarray analysis during embryogenesis (Figure 2A, see Additional file 5). The whole process was divided into two main sections in terms of hierarchical clustering of miRNA expression, with one clear boundary between day 2 and day 3 embryos and the remaining time-points.

**Figure 2:** **MiRNA expression patterns during silkworm embryonic development**. (A) Hierarchical clustering analysis of the expression of 36 miRNAs obtained from embryos of early 1^st ^instar larvae. The colors represent relative and mean-centered expression for each miRNA: green, low; black, mean; red, high. a and b represent the average signals of each probe printed at three points on each block. (B) Northern blotting analysis of miRNAs in the embryos and early 1^st ^instar larvae. 5srRNA and U6 served as the loading controls.

Small and large miRNA transcripts were detected in pre-laid eggs and embryos, and were identified as *miR-8*, *miR-252 *and *let-7 *(indicated with a red arrow in Figure 2B). Accumulating large fragments of these miRNAs suggest that maturation of functional small molecules involves sequential cleavage from larger transcripts [39]. Seven "early" miRNAs were detected in freshly deposited eggs (including *bantam*, *miR-92*, and *miR-184-3p*), which continued to be expressed until the formation of the synkaryon (6 h Em) (Additional file 5). Whole-life analysis revealed that *miR-92 *expression was restricted to three time-points during the course of development from embryo to moth, and peaked at the day 6 embryo stage (Additional file 4). A more precise examination disclosed a significantly extended existence during embryogenesis and a virtual expression peak in the day 3 embryo (Additional file 5). After fertilization, the synkaryon undergoes synchronous mitosis, resulting in the formation of blastoderm and the subsequent germband. Numerous cleavage nuclei begin to penetrate the periplasm about 10 h after oviposition. However, microarray and Northern blotting confirmed that few miRNAs were expressed at this time (12 h Em) (Figures 2A, B, Additional file 5), possibly because of the impending diapause stage [38]. After a further 12 h (24 h Em), 12 miRNAs were detected soon after egg release from diapause, including the 7 "early" miRNAs and others observed for the first time (miR-252, miR-8, miR-2a, miR-79, and miR-10b-3p). Expression of these miRNAs continued for 24 h (2 d Em), with slight fluctuations during the time of cell differentiation, to successively form the germband, amnion, gastrulation apparatus, and even the appendages of the abdomen and telson. One day later (3 d Em), expression of another group of miRNAs was initiated during the blastokinesis period after formation of the neural groove and abdominal appendages. In view of the finding that morphogenetic processes are severely affected in miRNA-devoid embryos [17], we propose that these miRNAs act concertedly to regulate the morphogenesis oforgans.

After blastokinesis, the embryo resumes growth by successively forming dorsal integument, the alimentary canal, setae, the epidermis, and the trachea, possibly involving several genes expressed during formation of larval organs [38]. This occurs around the head pigmentation stage in day 6 embryos. At this time-point, 8 miRNAs were initially expressed (including miR-29b, miR-34b, and miR-124). Once the larval organs form, the serosa is digested and pigmentation of the head and body progresses, but no other important morphological changes occur in the embryo [38]. However, a higher number of miRNAs were initially present in day 9 embryos (9 d Em) at the body pigmentation stage, including miR-281-5p, miR-281-3p, miR-263, miR-970, miR-133, miR-283, and miR-317. During the subsequent 24 h, the young larvae inside the eggshells eat and break the chorion around the micropylar region and emerge [38]. No distinct differences in miRNA expression existed between newly hatched silkworms and day 9 embryos.

### miRNA expression in silkworm larvae correlates with stage transitions

To further investigate the correlation between miRNA expression and stage transition, we sampled throughout the larval stages from newly hatched silkworm to late 3^rd ^molt larva (early larval stages), and early 4^th ^instar larva to late 5^th ^instar larva (late larval stages). Day 2 and day 9 embryos served as controls to ensure comparable results. Twenty unique miRNAs were highly expressed, as shown by microarray experiments, during the early larval stages, including 15 strongly detected miRNAs identified in the whole-life array (Additional file 6). Late 2^nd ^instar larvae expressed the largest number of miRNAs, among which 25 displayed peak levels at this time-point (Additional file 6). The whole-life array revealed exclusive miR-29 expression at the early 1^st ^instar and late 1^st ^molt larval stages. In fact, miR-29 was additionally expressed in late 1^st ^instar, late 2^nd ^instar, and late 3^rd ^molt larvae. miR-92 was absent from the early 1^st^, 2^nd^, and 3^rd ^instar larval stages, but highly expressed in late 1^st^, 2^nd^, and 3^rd ^instar larvae and late 1^st^, 2^nd^, and 3^rd ^molt larvae. The miR-124 level at the late 1^st ^instar larval stage was two-fold higher than that during the early 1^st ^instar larval stage. miR-124 was sharply up-regulated to peak levels from the time of its initial expression in the day 6 embryo, followed by down-regulation, despite waning in early 2^nd ^and early 3^rd ^instar larvae and early 3^rd ^molt larvae, and waxing in late 2^nd ^and late 3^rd ^instar larvae and late 3^rd ^molt larvae. In contrast, miR-100 and let-7 were initially expressed in late 2^nd ^instar larvae, and accumulated to high levels in late 3^rd ^molt larvae, with obvious fluctuations during the early larval stages. miR-34b and miR-275 exhibited complementary changes in patterns in whole-life profiling, but displayed sympathetic vibrations, particularly from the early 2^nd ^instar to late 3^rd ^molt stages, upon more detailed examination (Figure 3B). The presence of miRNAs during the early larval stages was further confirmed by Northern blotting (Figure 4A).

**Figure 3:** **Microarray analysis of miRNA expression during the larval stages**. (A) Stage-specifically expressed miRNAs during the early larval stages. (B) Comparison of the expression profiles of miR-275 and miR-34b during the early larval stages. (C) Stage-specifically expressed miRNAs during the late larval stages. (D) Comparison of miR-275 and miR-34b expression profiles during the late larval stages.

**Figure 4:** **Northern blotting analysis of miRNA expression during the larval stages**. (A) Northern blotting analysis of miRNAs during the early larval stages. (B) Northern blotting analysis of miRNAs during the late larval stages (C) A number of miRNAs displayed sex-dependent differences in expression at day 3 and day 7 fifth instar larval stages. 5srRNA and U6 served as the loading controls.

In total, 18 of the 20 miRNAs expressed throughout the early larval stages were maintained at high levels during late larval stages (Additional file 7). The two remaining miRNAs, miR-133 and miR-279, showed low levels of expression during the whole 4^th ^molt stage (Additional file 7). miR-100 and let-7 were up-regulated from 1^st ^instar to 3^rd ^molt, maintained over the 4^th ^and 5^th ^larval stages (Additional file 7), and highly expressed from early to late 4^th ^instar larvae and fifth-instar day 2 and day 7 larvae (Figure 3C). miR-274 displayed no expression signal during early larval stages, was initially detected in 5^th ^instar day 2 larvae, and was subsequently up-regulated to peak levels in day 7 larvae. miR-29b was detected at the late embryo and 1^st ^instar larval stages (Figure 3A), but was not expressed from early 4^th ^to 5^th ^instar day 7 larval stages (Additional file 7). miR-92 and miR-124 shared similar patterns with high expression at three time-points, specifically, late 4^th ^larval instar, and day 3 and day 7 5^th ^instar larvae, but was absent from 4^th ^molt larvae. The expression profiles of miR-275 and miR-34b were regulated in a complementary manner throughout the penultimate and final larval stages (Figure 3D). The changing expression profile of miR-275 by microarray was supported by Northern blotting results (Figure 4B). Some miRNAs displayed significant gender-specificity at the day 3 and day 7 fifth larval instar stages (Figure 4C), whereby signal values in females were at least two-fold higher than those in males.

The majority of expressed miRNAs oscillated with a clear-cut pattern corresponding to transitions between instar and molt stages, specifically, being higher at the late 1^st^, 2^nd^, and 3^rd ^instars and the late 3^rd ^molt, and lower at the early 1^st^, 2^nd^, and 3^rd ^instars and the early 3^rd ^molt (Additional file 8A). As with expression patterns at the early larval stages, most miRNAs exhibited a defined expression pattern during the 4^th ^and 5^th ^larval stages, specifically, up-regulation at the 4^th ^instar, down-regulation at the 4^th ^molt, up-regulation at the day 2 to day 3 fifth instar, down-regulation for 2 days, followed by a sharp increase again at day 7 (Additional file 8B). Interestingly, these coordinate expression changes were generally in keeping with ecdysone pulsing [40].

### Expression profiles of miRNAs in spinning larvae, pupae and moths

To determine the expression profiles of miRNAs at the spinning larva (Sp), pupa (Pu), and adult (Ad) stages, the whole-life test (Additional file 4) was applied from the development of the spinning larva to adult moth at 15 and 14 specific time-points for females and males, respectively. Based on hierarchical clustering, samples from the larval, pupal, and adult stages were clearly separated (Figure 5A). The proximal stages displayed similar miRNA expression profiles. Therefore, miRNA expression patterns may be applied as a developmental marker of silkworm individuals, as suggested for the developing mammalian brain [33]. In total, 15 miRNAs were highly expressed throughout pupal and adult stages by microarray, among which 10 were common to both sexes and 9 were robustly expressed over the whole life cycle (including miR-252, miR-1, and let-7a) (Additional files 9 and 10). A number of miRNAs were also confirmed in females by Northern blotting (let-7a, let-7b, miR-8, and miR-2a) (Figure 5B). Moreover, Northern blotting revealed the presence of miR-263b throughout the metamorphosis process, although high expression was only evident in day 6 and day 7 pupae in microarray experiments. In females, the 55 expressed miRNAs peaked at eight time-points (20 in the day 7 pupa and 10 in the egg-removed moth stage) whereas in males, the 52 expressed miRNAs displayed the highest signals at nine time-points (16 at early prepupal and 11 at day 4 pupal stages). However, specific miRNAs shared the same expression profile in both genders as larva-pupa-adult metamorphosis advanced, and expression of the majority of miRNAs abruptly fell at the day 3 pupa time-point (*see *Additional file 11). These results raise the issue of whether females and males share the same mechanism in coordinating miRNAs for the larval-pupa-adult transition. Illustratively, five miRNAs were compared between females and males (Figures 5C, D). In the whole-life test, miR-29b was not present in early female pupae, but was strongly expressed in the early female moth (Additional file 4). A more detailed examination revealed its initial expression in both genders at the day 4 pupal stage, and subsequent up-regulation. Whereas expression in both sexes fluctuated in a generally similar manner, miR-29b was far more highly expressed in females. The whole-life array revealed that, in contrast to miR-29b, miR-275 expression peaked in early female pupae, but not in the early female moth (Figures 1B, C). A precise test further revealed strongest expression in the prepupa and day 2 pupa in both females and males (Figures 5C, D). Moreover, both Northern blotting and microarray tests revealed down-regulation of miR-275 in both sexes during this process (Figure 5B, E). Unexpectedly, miR-275 was not expressed in the early female moth with eggs. However, when the eggs were manually removed from the maternal abdomen, miR-275 expression was significantly increased, further confirming its absence in pre-laid eggs and early embryo stages. Although the whole-life array did not confirm the existence of miR-274 in silkworms, the presence of this miRNA was verified in the fifth instar larva from days 2 to 7 (Figure 3C, Additional file 8). Interestingly, the detailed investigation revealed high expression in the spinning larvae of both genders, but no expression in pupae of either sex (Figure 5C, D, Additional files 9, 10), strongly implying an important function for this miRNA in the spinning activity of silkworms. miR-29b and miR-92 appeared to share similar patterns by whole-life profiling, but the detailed assay revealed evident differences between their expression profiles. miR-29b expression peaked in egg-removed moths, whereas miR-92 expression was maximal in the new pupae of both sexes. miR-34b was robustly expressed in females at the early cocoon spinning and new adult moth stages, but was expressed at only low levels in early pupae in the whole-life test (Figure 1, Additional file 4). Its expression in pupae and adults was further established by precise sampling (Figure 5C, D; Additional files 9, 10). miR-34b was not expressed, or was expressed at very low levels, in female pupae during the first 5 days, but was significantly up-regulated in day 6 pupa, and highly expressed in female adult moths with or without eggs. However, this miRNA was also nearly undetectable in the male prepupa and male pupae from 0 h to day 7, but displayed a sharp increase at day 8 and attained its highest expression in the fresh male adult moth, followed by an evident decrease 2 days later. The silkworm moth lives for only several days, and dies soon after mating or laying eggs. In keeping with the development of the silkworm body, the expression levels of all miRNAs in adults of both sexes decreased significantly within 2 days (Additional file 11).

**Figure 5:** **Profiling of miRNA expression during pupal metamorphosis**. (A) Developmental time-points were grouped using the hierarchical clustering method and gene sets from Additional file 9. Gene names and quantitative miRNA expression levels are presented in Additional file 9. (B) Northern blotting analysis of specific miRNAs in females. (C) Stage-regulated miRNAs in females. (D) Stage-regulated miRNAs in males. (E) Northern blotting analysis of specific miRNAs in males. Northern blots were exposed for different times, and thus the intensities of signals on one Northern blot cannot be directly compared to those from others. A probe against 5srRNA was hybridized to respective blots for comparison.

## Discussion

To the best of our knowledge, this is the first comprehensive investigation of miRNA expression profiles over the whole life-cycle of *Bombyx mori*. Although previous studies have examined four time-points representing the main developmental stages of the silkworm, to clarify the temporal expression profile of miRNAs [24-26], it is impossible to establish detailed expression patterns at stage transitions over the fifty-day life cycle with limited time measurements. The whole-life test used in the present study provided a general expression profile of miRNAs during silkworm development, and subsequent precise stage-by-stage examinations further confirmed the presence or absence of miRNAs at multiple time-points. The miRNAs exhibiting significant expression changes over the whole life cycle and specific developmental stages are summarized in Additional file 12. For example, the miR-10b-5p/3p pair was down-regulated in whole-life profiling, but stage-by-stage examination revealed up-regulation of these miRNAs during embryogenesis, followed by down-regulation during the early and late larval stages. Several miRNAs, such as miR-34b and miR-305, were up- or down-regulated in whole-life profiling, but in fact, displayed diverse or even opposite regulation patterns at some developmental stages.

Despite stable culture conditions of a 12 h light:12 h dark cycle, the temporal niche varies dramatically within the life-cycle of the silkworm, consequently exerting vital pressure on the capacity for temporal adjustment [41]. The Dazao silkworm is a bivoltine strain in which the nature of the diapause is dependent on incubation temperature. Specifically, incubation at 25°C produces only diapause eggs and incubation at 15°C produces exclusively non-diapause eggs [42]. Therefore, the temporal expression profiles of silkworm miRNAs may be under dual control of the developmental program and environmental stimuli, such as the polyprotein precursor mRNA, which is common to diapause hormone (DH) and pheromone biosynthesis activating neuropeptide (PBAN) [43]. In zebrafish, few miRNAs are expressed within 12 h post-fertilization. An increasing number of miRNAs are detected 1 to 2 days after fertilization and show strong expression when organogenesis is virtually complete [44]. In the early embryo of *Drosophila*, several miRNAs initiate expression at the onset of zygotic transcription [45]. Their dynamic expression patterns are mediated by tissue-specific enhancers [46]. In the silkworm, a small set of miRNAs weakly accumulated at fertilization (6h Em) or the early embryo stages (see Additional file 5). The maternal Dicer enables zygotic Dicer mutants of zebrafish to live for almost 2 weeks [9]. Emergence of these miRNAs in pre-laid or newly deposited eggs may also be attributed to maternal information, similar to the embryonic diapause induced by the diapause hormone (DH), which is secreted by the maternal subesophageal ganglion during pupal-adult development [43].

MiRNAs are absent in the zygotes of zebrafish, and are primarily detected during the blastula period [47]. The majority of zebrafish miRNAs are expressed in a tissue-specific manner during the late stage of embryonic development [44], and present widely divergent expression profiles throughout the 3 dpf and 5 dpf embryonic brain [48]. In frog (*Xenopus laevis*), an increasing number of miRNAs are expressed at specific stages as embryonic development proceeds, and are continuously expressed until the tadpole stage [49]. Few miRNAs are detected during the formation of primary germ layers of the chick, but rapid accumulation occurs during organogenesis [50]. Several miRNAs cannot be detected until the late specific stages of mouse (*Mus musculus*) embryonic development, but their transcription levels are markedly increased thereafter [51]. Overall, these data leave the intriguing question open as to whether and how these miRNAs are implicated in controlling the fate of protein-encoding genes during embryogenesis, consequently contributing to tissue differentiation and organogenesis.

During the prepupal and pupal stages of holometabolous insects, imaginal tissues and organs are newly formed from primordial cells and imaginal discs, whereas larval tissues degenerate in the pupa, and pupal tissues are fully lost in the adult [52]. Larval cuticles break down during the last day before pupal molt [53,54]. Oogenesis and ovarian development of *B. mori *are triggered by 20-hydroxyecdysone (20E) [55], and then pass through various stages for approximately 10 days from the fifth instar larvae to the pharate adult [56]. Hundreds of genes are required for the dramatic morphological changes in wing disc development during metamorphosis, although their intrinsic roles are yet to be established [57]. This *in vitro *progression is possibly controlled by unidentified non-coding RNAs [58]. Four miRNAs (miR-29b, miR-34b, miR-277, and miR-285) were significantly up-regulated from the spinning larvae to adult stages, and nine (miR-305, miR-275, miR-289, miR-307-3p, miR-274, miR-286, miR-87, miR-315, and miR-92) were significantly down-regulated during this time-course (Additional file 12). These opposite but coordinate expression changes during the non-feeding stages of females and males should pave the way for further analysis of the mechanisms underlying the metamorphosis of insects.

The normal formation of a mature insect egg is processed under concerted regulation of the steroid hormone ecdysone and its receptors [59-61]. Simultaneous expression of miR-125 and let-7 during *Drosophila *development is synchronized with the high- titer ecdysone pulses that initiate metamorphosis [62]. The ecdysone titer in silkworm fluctuates in response to stage transitions during embryogenesis [63], instar larval stages [40], and larval-pupal-adult development [64-66]. The majority of miRNAs are significantly up-regulated as the ecdysone synthesis rate rises at the end of each larval instar. Similarly, miRNAs are clearly down-regulated when ecdysone synthesis falls during the period from molt to instar larval stage. During pupal metamorphosis, several miRNAs were down-regulated in day 3 pupae of both sexes, consistent with a significant decrease in the ecdysone level. Thus, over the whole life cycle of silkworm, expression rhythms of several miRNAs may be coordinated by ecdysone. However, the miRNA expression profiles did not always fluctuate in accordance with the ecdysone titer. For example, miR-275 and miR-274 expression was typically stage-specific and unrelated to ecdysone pulsing. Furthermore, several miRNAs were upregulated at the end of the 3^rd ^and 4^th ^molt stages, presenting abnormal patterns in relation to ecdysone levels. Most miRNAs displayed two expression peaks at the 5^th ^instar larval stage (from day 2 to 3 and from day 5 to 7), whereas the ecdysone peaks on the last day of the 4^th ^instar larva rapidly declined at the early 4^th ^molt, and ecdysone was maintained at a low level until the onset of the wandering stage [65]. It is possible that additional factors, including hormones other than ecdysone, regulate miRNAs, as the expression rhythms were sometimes out of step with the ecdysone pulse.

## Conclusion

Here, we obtained initial temporal measurements of the levels of abundant miRNAs throughout the entire life-cycle of *Bombyx mori*. The diverse expression patterns of silkworm miRNAs strongly supports the idea that the miRNAs function at different levels to regulate silkworm development. Refined expression patterns corresponding to stage transitions may provide a strong molecular basis for further functional analysis of miRNAs in this animal model.

## Methods

### Computational prediction of silkworm miRNAs

We initially predicted silkworm miRNAs using miRscan algorithms, as described by Lim and colleagues [67,68], as well as homology searches with PatScan algorithms [69,70] with the first silkworm genome assembly (6× genome data) [71] and the limited number of miRNAs available in the miRBase release 4.0 [72]. The specific sequences that could form a correct hairpin structure (hairpin length larger than 55 bp and at least 6 base pairs in the arm) with low free energy (lower than -25 kcal/mol overall and lower than -0.27 kcal/mol per nucleotide) were submitted to microarray and Northern blotting analyses. Subsequently, we employed all the mature miRNAs from the miRNA repository miRBase 11.0 for a homology search for complementary sites on the silkworm genome with no more than 3 mismatches. Hits were extended on the genome and further filtered by limits based on the folding parameters determined by RNAfold [73,74] and mfold [75]. According to the current nomenclature guidelines [76-78], abbreviated 3 letter prefixes 'bmo' are used to designate the species of *B. mori*, mature sequences and precursor hairpins are labeled 'miR' and 'mir', respectively, and the different miRNA sequences excised from opposite arms of the same hairpin precursor are currently given names ending with -5p or -3p to distinguish the arms.

### Silkworm culture and RNA extraction

Female moths of the domesticated silkworm (*B. mori*), Dazao, were allowed to lay eggs for 4 h at 25°C. Developing eggs were incubated at 25°C from oviposition until hatching, the first day being the day of oviposition. When developing eggs were incubated at 25°C, head pigmentation occurred on day 7 (6 × 24 h after oviposition), body pigmentation appeared on day 9 (8 × 24 h after oviposition), and more than 95% of eggs hatched on the tenth day. To prevent entry into diapause, fertilized eggs were treated with a hydrochloric acid solution (4 N) at 46°C for 6 minutes and then rinsed thoroughly with water. After hatching, silkworm larvae were reared on mulberry leaves at 25°C and 85% H.R. under a 12 h light/12 h dark photoperiod, and harvested at the desired developmental stages. To obtain populations of *B. mori *at various developmental stages, animals were synchronized after oviposition by means of cold storage and acid treatment, keeping the diapause eggs at 4°C for at least three months, followed by 5 min of treatment with hydrochloric acid solution at 46°C. Moreover, developmental landmarks, including hatching, larval molting, mounting, spinning, pupariation and eclosion, were employed for more precise staging. Total RNA was extracted with TRIzol reagent (Invitrogen, Gaithersburg, MD), according to the manufacturer's instructions.

### Microarray printing and hybridization

The miRNA probes (denoted 'SW' followed by a serial number) on the microarray were designed to be complementary to the mature sequences of miRNAs, concatenated up to 40 nt with polyT, and modified with an amino group at the 5'-end. Since probe sets for some miRNAs are present more than once on the array, 106 probes for 92 unique miRNAs were used to establish the existence and profiling of miRNAs in the silkworm (Additional file 2). These comprised 45 probes for the homology-found miRNAs, 2 for special silkworm miRNAs, 4 for the antisense strands of miRNAs, 42 for miRNAs of other organisms, and 13 as replicate probes for several miRNAs. All probes, including the controls, were synthesized at MWG Biotech (Ebersberg, Germany), dissolved in EasyArray spotting solution (CapitalBio, Beijing, China) at a concentration of 40 μmol/L, and printed in triplicate on aldehyde-coated slides (CapitalBio) using a SmartArray-136 spotter (CapitalBio). Low molecular weight RNA (4 μg) isolated using PEG solution precipitation was labeled with fluorescent Cy3 using T4 RNA ligase, according to a previous protocol [79], and hybridized overnight to the microarray in 16 μl hybridization buffer (15% formamide, 0.2% SDS, 3×SSC, 50×Denhardt's) at 42°C. Following hybridization, slides were washed in a SlideWasher-8 instrument (CapitalBio) using washing bufferI (0.2%SDS, 2×SSC) and bufferII (0.2×SSC) and dried. Slides were scanned using a laser confocal scanner, LuxScan 10K-A, and images extracted using LuxScan 3.0 software (CapitalBio). Net signals were calculated by subtracting the local background from total intensities and spots with a negative signal awarded the value 10. To make the inter-slide signals comparable, signals were normalized using a global median method. Flaw spots were excluded for further analysis after visual inspection of the hybridization figures using a self-developed program, "Flaw-Spot-Finder", according to X and Y axes of the spot position on the array. Differentially expressed miRNAs were selected with Significance Analysis of Microarrays (SAM, version 3.0), as described previously [80,81]. The signal values of triplicate spots for each probe on individual slides were averaged, and individual samples hybridized with two replicate slides (indicated as lowercase a and b). The mean signal values were log_2 _transformed before submission to Gene cluster 2.0 for SOM analysis and Gene Cluster 3.0 for cluster analysis. Microarray data passing the threshold 1,000 were generally confirmed by Northern blotting. A signal value of 1,000 was set as the positive expression threshold.

### Northern blotting

Blots were prepared by electrophoresing 150 μg of total RNA per lane on a denaturing 12% polyacryamide-7 mol/l urea gel at 200 V for 1 h and 300 V for 2 h, followed by electroblotting to Hybond-N nylon membranes (Ambion) using the semi-dry Trans-Blot Electrophoretic Transfer cell (Bio-Rad). After electroblotting, RNAs were fixed to the membrane by UV cross-linking (1000 μJ, HL-2000 HybriLinker; UVP), followed by baking in a vacuum oven at 80°C for 30 min. DNA oligonucleotides complementary to the predicted candidate miRNAs, U6 RNA and 5srRNA were synthesized (Sangon, Shanghai). The 5'-ends of DNA and Decade Markers (Ambion) were labeled with [γ-^32^P] ATP (Amersham) using T4 polynucleotide kinase (Takara), and subjected to purification using a Purification Cartridge (Ambion). The membrane was pre-hybridized in solution containing 6×SSC, 10×Denhardt's solution, 0.2% SDS and 50 μg salmon sperm DNA (Ambion) at 65°C for about 5 h. Membranes were hybridized in solution containing 6×SSC, 5×Denhardt's solution, 0.2% SDS and 50 μg denatured sheared salmon sperm DNA (Ambion) with 1-5 × 10^6 ^cpm eluted radiolabeled oligonucleotide probes at 10-15°C below the calculated dissociation temperature for at least 10 h. Blots were washed three times for 5 min each at 37°C with 6×SSC and 0.2% SDS, and once at 42°C for at least 15 min. After the final wash, blots were wrapped in plastic film and exposed to X-ray film at -70°C for 24 to 72 hours. The former probe was stripped for reprobing by washing at 90°C in 0.1×SSC, 0.5% SDS. Radioactive signals were quantified with the ImageQuant software package (Molecular Dynamics).

## Abbreviations

0 h Em: 0 hour embryo; 6 h Em: 6-hour embryo; 12 h Em: 12-hour embryo; 24 h Em: 24-hour embryo; 2 dEm: day 2 embryo; 3 dEm: day 3 embryo; 6 d Em: day 6 embryo; 9 dEm: day 9 embryo; eIL1 (0 h IL1): early 1^st ^instar larva; lIL1: late 1^st ^instar larva; lML1: late 1^st ^molt larva; eIL2: early 2^nd ^instar larva; lIL2: late 2^nd ^instar larva; lML2: late 2^nd ^molt larva; eIL3: early 3^rd ^instar larva; lIL3: late 3^rd ^instar larva; eML3: early 3^rd ^molt larva; lML3: late 3^rd ^molt larva; eIL4: early 4^th ^instar larva; lIL4: late 4^th ^instar larva; eML4: early 4^th ^molt larva; lML4: late 4^th ^molt larva; eIL5: early 5^th ^instar larva; 2 dIL5: fifth-instar day 2 larva; 3 dIL5 (f): female fifth-instar day 3 larva; 3 dIL5 (m): male fifth-instar day 3 larva; 5 dIL5 (f): female fifth-instar day 5 larva; 5 dIL5 (m): male fifth-instar day 5 larva; 5 dIL7 (f): female fifth-instar day *7 *larva; 5dIL7 (m): male fifth-instar day *7 *larva; efSp (0 h fSp): early female cocoon-spinning larvae; 0hPPu: early prepupa; efPu (0 h fPu): early female pupa; efAd (0 h fAd): early female adult; 0 h Ad (EB): fresh adult moth with eggs in its abdomen (0-hour egg-bearing adult moth); 0 hAd (ER): fresh adult moth whose eggs were manually removed (0-hour egg-removed adult moth); 2 dAd (EL): day 2 adult moth after laying eggs (day 2 egg-laid adult moth).

## Authors' contributions

SL conceived and designed the study, performed microarray and Northern blotting hybridization experiments, analyzed data, and wrote the manuscript. QX, PZ and ZX coordinated the study. QL performed miRNA prediction and analysis. LZ, DC and JD performed microarray experiments and generated array data. QX reviewed the manuscript. All authors read and approved the final manuscript.

## Supplementary Material

Additional file 1 **microRNAs examined in this study**. (A) miRNAs subjected to homology searches and two silkworm-specific miRNAs. This set of conserved miRNAs comprised the majority of silkworm miRNAs subjected to homology searches due to the expanding miRBase. Therefore, some miRNAs were not probed in this microarray (such as let-7b). 'SW' followed by a number represents the serial number of one probe printed on the microarray slides. 'Homologs' column includes the corresponding names of miRNAs of other organisms. The 'location' column depicts the genome site of the mature sequence (left) and the precursor (right). The loci of miRNAs were described in the 'locus description' column. The 'arm' column shows that the mature sequence originates from either arm of the precursor. The folding energy of the stem-loop structure is presented on the 'dG' column. Most miRNAs found by homology searches can be localized on the chromosomes ('chr.' Column). The 'str.' column shows the sense or antisense strand encoding miRNAs. (B) Specific antisense sequences were probed to determine their presence or absence. anti-miR-276-5p, anti-miR-124 and anti-miR-263b displayed signals higher than the threshold of 1,000 at the late 3^rd ^molt and 4^th ^molt stages. Moreover, anti-miR-276-5p displayed signals above 1,000 in day 3 fifth instar larva and day 6 female pupa as well as at three time-points of male pupa. These findings suggest that antisense transcriptions of some miRNAs also exist in silkworm. (C) Alternative strands of specific miRNAs. Alternative forms were probed independently as repeats to ascertain whether results were reproducible. Alternative probes of the specific miRNAs clearly yielded identical results (let-7a and let-7a#; miR-275 and miR-275#). (D) miRNAs from other organisms. A large number of miRNAs are highly conserved between species. However, only a few match the primary silkworm genome data. Accordingly, we also probed 42 miRNAs of other organisms. Remarkably, nearly half of these were confirmed using both Northern blotting and microarray. In this table, names, mature sequences, homolog miRNAs, locus description, arm, folding energy (dG, Kcal/mol), chromosome (chr) are shown, and supplementary information is excluded due to limited space. Click here for file

Additional file 2 **Printing design and oligonucleotides for the miRNA microarray chip**. This table presents the probe location on the microarray slide. 'Bock' represents the microarray slide with all printed probes. To obtain convincing results, all probes for miRNAs and controls were printed in triplicate on two parallel blocks. Moreover, a number of time-points were repeatedly sampled and examined with the microarray blocks. Numbers presented in 'Row' and 'Column' represent the loading site on each block. 'ID' is the respective locus for each printing. 'Oligo name' is the probe ID. Click here for file

Additional file 3 **Whole-life test on miRNA expression in the silkworm by Northern blot hybridization**. To obtain general whole-life expression patterns of miRNAs in the silkworm, we performed Northern blot hybridization. 5srRNA and U6 were used as the loading controls. Abbreviations: 6 d Em, day 6 embryo; eIL1, early 1st instar larva; lML1, late 1st molt larva; eIL2, early 2nd instar larva; lML2, late 2nd molt larva; eIL3, early 3rd instar larva; eML3, early 3rd molt larva; eIL4, early 4th instar larva; eML4, early 4th molt larva; eIL5, early 5th instar larva; efSp (0 h fSp), early cocoon-spinning larvae; efPu (0 h fPu), early female pupa; efAd (0 h fAd), early female adult. Click here for file

Additional file 4 **Identification of miRNAs over the whole life cycle of silkworms**. A normalized signal value ≥ 1,000 was considered the positive expression threshold. +, expressed; -, not expressed. #, some miRNAs were hybridized to more than one probe containing several nucleotides more or less at the ends. 15 unique miRNAs were detected at all developmental stages. peak, the highest signal value on microarray. Nor., summarized Northern blot results; reg. regulation types; up, up-regulated expression; down, down-regulated expression NA, not assayed. Click here for file

Additional file 5 **Identification of miRNAs during embryogenesis by microarray**. In total, 36 unique miRNAs were selected as 'expressed' during embryogenesis. +, expressed; -, not expressed; peak, the highest expression level obtained from this test; the 'points' column depicts the total positive time-points; the 'WLE' column shows whole-life expression with the general whole-life test; 'SUM' row represents the total number of expressed unique miRNAs at a specific time-point; E6-, not detected in day 6 embryo with the whole-life test. Abbreviations: 0 h Em, 0 hour embryo; 6 h Em, 6-hour embryo; 12 h Em, 12-hour embryo; 24 h Em, 24-hour embryo; 2 dEm, day 2 embryo; 3 dEm, day 3 embryo; 6 dEm, day 6 embryo; 9 dEm, day 9 embryo; 0 h IL1(eIL1), early 1st instar larva. Click here for file

Additional file 6 **Identification of miRNAs by microarray during the early larval stages**. In total, 62 unique miRNAs were selected as 'expressed' during the early larval stages, of which 23 were not detected in the whole-life test. Twenty unique miRNAs displayed expression signals above the threshold in all the time-points examined from day 9 embryo to late 3rd molt. +, expressed; -, not expressed; peak, highest expression level obtained with this test; the 'points' column presents the total positive time-points; WLE, whole-life expression with the general whole-life test; 'SUM' row represents the total number of expressed unique miRNAs at a specific time-point; E6-, not detected in day 6 embryo with the whole-life test. Abbreviations: 2 d Em, day 2 embryo; 9 d Em, day 9 embryo; eIL1, early 1st instar larva; lIL1, late 1st instar larva; lML1, late 1st molt larva; eIL2, early 2nd instar larva; lIL2, late 2nd instar larva; lML2, late molt larva; eIL3, early 3rd instar larva; lIL3, late 3rd instar larva; eML3, early 3rd molt larva; lML3, late 3rd molt larva. Click here for file

Additional file 7 **Identification of miRNAs by microarray during the late larval stages**. In total, 54 unique miRNAs were selected as 'expressed' during the late larval stages, among which 16 were not detected with the whole-life test. Twenty unique miRNAs displayed expression signals above the threshold at all the time-points examined from early 4th instar larva to fifth-instar day 7 larva. +, expressed; -, not expressed; peak, highest expression level obtained with this test; the 'points' column shows the total positive time-points. 'eIL' column presents miRNAs expressed throughout the early larval stages; 'WLE' column shows whole-life expression with the general whole-life test; 'SUM' row is the total number of expressed unique miRNAs at a specific time-point; E6-, not detected in day 6 embryo with the whole-life test. Abbreviations: eIL4, early 4th instar larva; lIL4, late 4th instar larva; eML4, early 4th molt larva; lML4, late 4th molt larva; eIL5, early 5th instar larva; 2dIL5, fifth-instar day 2 larva; 3dIL5(f), female fifth-instar day 3 larva; 3dIL5(m), male fifth-instar day 3 larva; 5dIL5(f), female fifth-instar day 5 larva; 5dIL5(m), male fifth-instar day 5 larva; 5dIL7(f), female fifth-instar day 7 larva; 5dIL7(m), male fifth-instar day 7 larva. Click here for file

Additional file 8 **Microarray-based expression levels of miRNAs correlate with stage transitions of larvae**. (A) Fluctuating miRNA expression corresponding to stage transitions during the early larval stages. (B) Fluctuating miRNA expression corresponding to stage transitions during the late larval stages. The colors indicate relative and mean-centered expression for each miRNA: green, low; black, mean; red, high. The lowercase letters a and b represent the average signals of each probe printed at three points on individual blocks. Abbreviations of the samples are described in the figure legends to Additional files 6 and 7. Click here for file

Additional file 9 **Identification of miRNAs in the female silkworms from spinning to adult stages with microarray**. In total, 55 unique miRNAs were screened as expressed miRNAs in females across spinning larva, pupa and adult, among which 16 were not detected using the whole-life test. At all examined time-points across these stages, 15 unique miRNAs displayed expression signals above the threshold, and 10 were also expressed throughout in males. Clearly, day 3 pupae expressed the lowest and day 7 pupa expressed the highest number of miRNAs. +, expressed; -, not expressed; peak, Highest expression obtained with this test; the 'points' column depicts the total positive time-points; 'male' column depicts miRNAs expressed in males throughout these stages; 'WLE' column presents whole-life expression patterns obtained using the general whole-life test; 'SUM' row is the total number of expressed unique miRNAs at a specific time-point; E6 -, not detected in day 6 embryo with the whole-life test. Abbreviations: 0 hSp, early spinning larva; 0 hPPu, early prepupa; 0 hPu, early pupa; 12 hPu, 12-hour pupa; 24 hPu, day 1 or 24-hour pupa; 2 dPu, day 2 pupa, 3 dPu, day 3 pupa; 4 dPu, day 4 pupa; 5 dPu, day 5 pupa; 6 dPu, day 6 pupa; 7 dPu, day 7 pupa; 8 dPu, day 8 pupa; 0 hAd(EB), fresh adult moth with eggs in its abdomen; 0 hAd(ER), fresh adult moth whose eggs were manually removed; 2 dAd(EL), day 2 adult moth after laying eggs. Click here for file

Additional file 10 **Identification of miRNAs expressed by microarray in male silkworms from spinning to adult stages**. Overall, 54 unique miRNAs were selected as 'expressed' miRNAs in males across spinning larva, pupa and adult. Among these, 12 were not detected with the whole-life test. In total, 13 unique miRNAs displayed expression signals above the threshold at all the time-points examined across the stages, and 10 were additionally expressed throughout all stages in females. Similar to females, day 3 pupa expressed the lowest, while day 4 pupa expressed the highest number of miRNAs. +, expressed; -, not expressed; peak, highest expression level obtained with this test; the 'points' column presents the total positive time-points; 'female' column shows miRNAs expressed in females throughout these stages; 'WLE' presents the whole-life expression patterns obtained with the general whole-life test; 'SUM row is the total number of expressed unique miRNAs at a specific time-point; E6-, not detected in day 6 embryo with the whole-life test. Abbreviations: 0 hSp, early spinning larva; 0 hPPu, early prepupa; 0 hPu, early pupa; 12 hPu, 12-hour pupa; 24 hPu, day 1 or 24-hour pupa; 2 dPu, day 2 pupa, 3 dPu, day 3 pupa; 4 dPu, day 4 pupa; 5 dPu, day 5 pupa; 6 dPu, day 6 pupa; 7 dPu, day 7 pupa; 8 dPu, day 8 pupa; 0 hAd, fresh adult moth; 2 dAd, day 2 adult moth. Click here for file

Additional file 11 **Microarray-based expression of miRNAs in spinning larvae, pupae and adults**. (A) Fluctuating expression levels in female silkworms during pupal metamorphosis. (B) Fluctuating expression levels in male silkworms during pupal metamorphosis. Both females and males displayed a deep expression trough at the day 3 pupa stage for the majority of miRNAs (indicated with red arrows). Abbreviations are described in the figure legends to Additional files 9 and 10, respectively. Click here for file

Additional file 12 **miRNAs are regulated in multiple ways during silkworm development**. All microarray data were analyzed using SAM 3.0. The miRNAs presented are specifically up- or down-regulated in the whole-life test or stage-by-stage assay. Early larvae comprise the 1st, 2nd and 3rd stages, while late larvae comprise the 4th and 5th stages. Sp-Pu-Ad (f)/(m), from spinning larvae to pupae and adults (females or males); reg, regulated; score (d), the T-statistic value; up, up-regulated; down, down-regulated. Click here for file
